# Identification of Drug-Disease Associations Using a Random Walk with Restart Method and Supervised Learning

**DOI:** 10.1155/2022/7035634

**Published:** 2022-10-10

**Authors:** Xiaoqing Liu, Wenjing Yi, Baohang Xi, Qi Dai

**Affiliations:** ^1^College of Sciences, Hangzhou Dianzi University, Hangzhou 310018, China; ^2^College of Life Sciences, Zhejiang Sci-Tech University, Hangzhou 310018, China

## Abstract

Drug-disease correlations play an important role in revealing the mechanism of disease, finding new indications of available drugs, or drug repositioning. A variety of computational approaches were proposed to find drug-disease correlations and achieve good performances. However, these methods used a variety of network information, but integrated networks were rarely used. In addition, the role of known drug-disease association data has not been fully played. In this work, we designed a combination algorithm of random walk and supervised learning to find the drug-disease correlations. We used an integrated network to update the model and selected a gene set as the start of random walk based on the known drug-disease correlations data. The experimental results show that the proposed method can effectively find the correlation between drugs and diseases, and the prediction accuracy is 82.7%. We found that there are 8 pairs of drug-disease relationships that have not yet been reported, and 5 of them have pharmacodynamic effects on Parkinson's disease. We also found that a key linkage between Parkinson's disease and phenylhexol, a drug for the treatment of Parkinson's disease *α*-synuclein and tau protein, provides a useful exploration for the effectiveness of the treatment of Parkinson's disease.

## 1. Introduction

With the prevalence of complex diseases, the existing drugs are far from meeting the needs of human beings to fight against diseases. At the same time, due to the rising cost of drug research and development, long research and development cycle, large difference in research and development success rate, and high loss rate of new drugs, the research and development of innovative drugs has become a major challenge in the medical field.

At present, reusing compounds that have reduced risk to treat common or rare diseases has become a popular means of drug research and development. This strategy is called drug repositioning or drug reuse. This method not only reduces the overall development cost but also shortens a large amount of research and development time [1–3]. Through drug repositioning, pharmaceutical companies have achieved many successes, such as Pfizer's Viagra for erectile dysfunction [4] and Celgene's thalidomide for severe nodular leprosy erythema [5].

With the rapid expansion of large-scale genome, transcriptome and proteome data, computational drug repositioning study has emerged as one of the leading methods. Huang et al. developed a new drug repositioning pipeline to analyze four lung cancer microarray datasets, enrich biological processes, potential therapeutic drugs, and target genes for the treatment of non-small-cell lung cancer (NSCLC) [6]. They integrated two methods: machine learning algorithm and classification based on topological parameters. Zheng et al. designed a weighted ensemble similarity (WES) algorithm which provides a new perspective for drug repositioning and discovery [7]. Wang et al. integrated two drug transfer methods and proposed a new method for drug repositioning [8]. Cheng et al. [9] integrated the integration of chemical, gene, and disease networks, inferred the chemical hazard profile, studied the exposure data gap, and fully considered the gene and disease network in the chemical safety assessment [10]. A large number of genetic and molecular biology studies have shown that diseases reflect the interaction of multiple molecular components on a certain level [11–14]. Therefore, drug repositioning study should consider the interaction between different disease-related genes [15–18]. Luo et al. found the potential indications of a given drug based on some comprehensive similarity measures and Bi-Random walk (BiRW) [19]. Yu et al. inferred the correlation between drugs and diseases by studying the characteristics of known protein complexes [20]. PREDICT (PREdicting Drug IndiCaTions) considers that similar drugs are suitable for similar diseases; the prediction task is achieved by designing similarity measures between multiple drugs and diseases [21].

The above method was successfully applied to drug-disease association study and achieved good performance. However, these methods have used a variety of network information, but the integrated network is still less used. With the increase of the related data of known drug diseases, a supervised learning method should be designed to further improve the drug-disease association research by using the related data of known drug diseases. In this paper, we used an integrated network consisting of HPRD, BioGRID, STRING, and other databases. Unlike previous network-based studies, which used the random walk method with restart on the network, we updated the model using the known data of the relationship between drugs and diseases and selected a gene set as the starting point of random walk, thus realizing the supervised learning of random walk with restart method. We also evaluated the performance of the proposed methods in various diseases and analyzed their GO and KEGG function enrichment.

## 2. Datasets and Methods

### 2.1. Protein–Protein Interaction (PPI) Network

Human protein–protein interaction (PPI) network is selected, which has been compiled by Jörg et al. that contained experimentally documented human physical interactions from TRANSFAC, IntAct39, MINT40, BioGRID41, HPRD42, KEGG43, BIGG44, CORUM45, PhosphoSitePlus46, and a large scale signaling network47. We used the largest connected component of the interaction in our analysis, consisting of 141,150 interactions between 13,329 proteins. Entrez Gene IDs were used to map disease-associated genes to the corresponding proteins in the interaction. The interaction and disease-gene association data is provided as a supplementary data set in Menche et al. [22]

### 2.2. Disease and Disease-Gene Data

Medical Subject Headings (MeSH) is an authoritative thesaurus compiled by the National Medical Library of the United States [23]. The disease subject words in the vocabulary provided by MeSH have perfect vocabulary classification. Our disease data and drug data are derived from Menche et al. [22], which integrate some genetic disease-related genes from the human Mendelian inheritance in man (OMIM: Online Mendelian Inheritance in Man) and trait gene association data from GWAS central. Through the medical topic title Ontology (MeSH) [24], the disease names of different disease nomenclature are combined into one name.

We screened diseases containing at least 20 disease-related genes from 1489 diseases in MeSH. In this paper, we considered at least 20 disease-related genes in order to understand the role of related genes in the interaction network, rather than the occurrence of disease due to the mutation of a gene. Finally, 299 diseases and their 3173 genes were obtained. In the process of disease screening, we required at least one drug for each disease. By searching the DrugBank database, the drug information that can treat 79 diseases corresponding to FDA approval is obtained, and Metab2Mesh is used for text mining [25]. If the text mining results indicate that there is a strong correlation between disease and drug, we added the relationship between the drug and disease into the known data set.

### 2.3. Drug and Drug-Target Data

DrugBank is a comprehensive drug information database, which not only includes the information of drug structure, drug target, and drug action mechanism but also integrates the information of drug experiment and clinical research. DrugBank has strong retrievable ability, coupled with its convenient web visualization function, which provides researchers with powerful convenience in drug research and development, drug mechanism exploration, and so on. DrugBank 5.0 contains information about 10971 drugs and 4900 protein targets, including 2391 FDA approved small molecule drugs, 934 approved biotechnology drugs, 109 nutritional drugs, and more than 5090 experimental drugs. We collected the drug and drug-target information certified by the FDA from DrugBank, and then searched for the strong literature evidence of drug-early-warning-disease association through Metab2Mesh, and finally obtained 238 drugs that can treat corresponding diseases.

### 2.4. Random Walk with Restart Method

PPI network can be expressed as *G* = (*V*, *E*), where *V* denotes protein and *E* stands for protein–protein interaction. The *n*∗*n* adjacency matrix *A* is used to represent the PPI network, where *n* is the total number of the proteins. If there is interaction between protein *i* and protein *j*, *A*_[*i*, *j*]_ is 1, otherwise it is 0. We then normalized the adjacency matrix *A*:

(1) $$\begin{array}{c} A_{\left[i,j\right]}^{\prime }=\frac{A_{\left[i,j\right]}}{\sum_{k=1}^{n}A_{\left[k,j\right]}}. \end{array}$$

Random walk is used to find potential gene association data of diseases or drugs. When the random walk converges, the probability of a disease or drug at each point of the PPI network can be obtained. The relationship between drugs and diseases can be calculated based on the correlation between the probability distribution of diseases and drugs.

Random walk starts with a set of seed genes. The initial vector of seed genes is defined as follows:

(2) $$\begin{array}{c} P_{0}={\left[\psi_{1},\psi_{2},\cdots ,\psi_{n}\right]}^{T}. \end{array}$$

For a disease, we listed all the drugs that can treat it, incorporate all the genes of these drugs into the relevant genes of the disease, and took the combined gene set as the seed gene of the disease. Among them, the genes directly related to the disease are defined as

(3) $$\begin{array}{c} P_{{\text{dis}}_{\text{dir}}}=\left[\psi_{{\text{dis}}_{{\text{dir}}_{1}}},\psi_{{\text{dis}}_{{\text{dir}}_{2}}},\cdots ,\psi_{{\text{dis}}_{{\text{dir}}_{\text{n}}}}\right]{,}^{T} \end{array}$$

where the disease-related genes *ψ*_dis_dir_i___ will be set to 1, otherwise it will be set to 0. Then *P*_dis_dir__ is normalized as

(4) $$\begin{array}{c} P_{{\text{dis}}_{{\text{dir}}_{k}}}^{\text{‘}}=\frac{P_{{\text{dis}}_{{\text{dir}}_{k}}}}{\sum_{k=1}^{n}P_{{\text{dis}}_{{\text{dir}}_{k}}}}. \end{array}$$

Suppose there are *m* drugs that can treat the same disease, they are represented as  *P*_dis_drug_1___, *P*_dis_drug_2___, ⋯, and *P*_dis_drug_*m*___

(5) $$\begin{array}{c} P_{{\text{dis}}_{{\text{drug}}_{m}}}={\left[\psi_{{\text{dis}}_{{\text{drug}}_{m_{1}}}},\psi_{{\text{dis}}_{{\text{drug}}_{m_{2}}}},\cdots ,\psi_{{\text{dis}}_{{\text{drug}}_{m_{n}}}}\right]}^{T}. \end{array}$$

Sum all drugs for a disease:

(6) $$\begin{array}{c} P_{\text{di}{\text{s}}_{\text{drug}}}=\overset{m}{\underset{k=1}{\sum }}P_{\text{di}{\text{s}}_{{\text{drug}}_{k}}}. \end{array}$$

Then we normalized *P*_dis_drug__ as

(7) $$\begin{array}{c} P_{\text{di}{\text{s}}_{{\text{drug}}_{k}}}^{\text{‘}}=\frac{P_{\text{di}{\text{s}}_{{\text{drug}}_{k}}}}{\sum_{k=1}^{n}P_{\text{di}{\text{s}}_{{\text{drug}}_{k}}}}. \end{array}$$

Finally we got its seed gene for a given disease,

(8) $$\begin{array}{c} P_{\text{disease}}=tP_{{\text{dis}}_{\text{dir}}}^{\text{‘}}+\left(1-t\right)P_{{\text{dis}}_{\text{drug}}}^{\text{‘}}, \end{array}$$

where *t* is 0.5.

We also got the seed gene *P*_drug_ of a given drug following the same method. Start random walk and randomly access adjacent genes in each time scale (*t*⟶*t* + 1), the state probability *P*_*t*+1_ at time *t* + 1is

(9) $$\begin{array}{c} P_{t+1}=\left(1-r\right)A^{\prime }P_{t}+rP_{0}, \end{array}$$

where *P*_0_ is the initial vector, *P*_*t*_ is the probabilities at time *t*, and *r* is the restart probability. If the difference between *P*_*t*_ and *P*_*t*+1_ is less than 1*e* − 6, it is considered that the process will reach a stable state. After reaching the stable state, the correlation between drugs and diseases, drugs and drugs, and diseases and diseases is calculated according to the probability of drugs and diseases accessing each node on the network.

### 2.5. Supervised Learning

Cross-validation is a frequently used model validation technology. It divides the known data into two subsets, adds the data of one subset to the model training, and verifies the model with the remaining subset to evaluate the performance of the model in unknown data. For example, when using *k*-fold cross validation, the known data set needs to be randomly divided into *k* parts. In each cross-validation, *k*-1 data is selected to be added to the model training, and the remaining data is used for validation. Repeat for *k* times and select one piece of data for verification each time until each piece of data is tested.

The goal of cross-validation is to test the prediction ability of the model in new data, and it can also reflect the problem of overfitting or selection bias. In this paper, the idea of this method is used for supervised learning of random walk. For a certain disease, all drugs that can treat the disease in the data set are listed, and the genes associated with these drugs are incorporated into the relevant genes of the disease, and the combined gene set is used as the start of random walk. Needles are treated in the same way as drugs. In this paper, 403 known drug-disease associations between 78 diseases and 238 drugs were randomly divided into 10 parts. Nine of the disease and drug association data were selected to update the model, and the updated model was used to process the other data, so as to achieve the effect of supervised learning.

### 2.6. Evaluation Method

Receiver operating characteristic (ROC) curve is a curve based on the true positive rate (TPR) and false positive ratio (FPR) under various threshold settings. Area under the curve of ROC, also known as AUC value, can well reflect the performance of the classifier. The value of AUC varies between 0 and 1. When the AUC value is equal to 0.5, it means that the classifier cannot work. The larger the AUC value, the better the performance of the classifier. When the AUC value is 1, the classifier can produce perfect results.

## 3. Results

### 3.1. Performance Evaluation of the Random Walk with Restart Method Based on Supervised Learning

In order to evaluate the effectiveness of the proposed method, we first took the known drug-disease association as an independent validation data set. According to the relevant genes of 78 diseases and the drug targets of 238 drugs, the correlation information between diseases and drugs was obtained through restart random walk on PPI network. According to the ranking of drug-disease information pair by correlation, the AUC value was calculated. Three PPI networks BioGrid, HPRD, and STRING were independently verified, and their AUC results were 0.64, 0.52, and 0.66.

In order to further explore the efficiency of methods in different diseases, MeSH was used to classify all diseases. There are also some diseases in the classification that belong to a variety of disease types, such as colorectal tumors, which belong to C04 tumor diseases and C06 digestive system diseases. For the above case, we only calculated the average AUC value according to one of them. The AUC value was calculated on the basis of PPI network and optimal parameters. The classification results of various diseases are shown in Table 1.

From Table 1, it is easy to note that the performance of the random walk with the restart method is different among various diseases. It achieves good performance in the diseases of blood and lymphatic system C15, endocrine system diseases C19, eye diseases C11, and Male genitourinary system C12, with AUC values above 0.8. The highest is blood and lymphatic system C15, with an AUC value of 0.877. The AUC value of nervous system diseases is low, only 0.62.

In order to further verify the efficiency of the random walk with the restart method and supervised learning, we randomly divided all known drug-disease relationships into ten parts, nine pieces of data are used as the training set and the other is used to calculate AUC. For a certain disease, we listed all the drugs that can treat the disease in the known training set, and then integrated all the related genes of these drugs into the related genes of the disease, and took the combined gene set as the start of random walk [26]. For drugs, the same method is used; that is, the relevant genes of diseases that can be treated by a drug in the training set were combined into the target information of the drug. Ten AUC values were obtained for each experiment. In order to reduce random interference, the above experiment was repeated 10 times, and a total of 100 AUC values were obtained, as shown in Figure 1.

The results show that the average value of 100 AUC values is 0.827, indicating that the proposed method found the relationship between drugs and diseases. With the help of the training data of the known network relationship between drugs and diseases, the prediction sensitivity of drugs and diseases was further improved. Adding the target information of drugs that can treat a disease to the disease-gene information will indirectly add some potential disease-gene information, making the disease-gene information more abundant. Similarly, adding the genes of all diseases that can be treated by a drug to the target information of drugs can also enrich the information of drug-action targets and make the relationship between drugs and diseases more discovered, thus improving the prediction of drug sensitivity.

### 3.2. Analysis of the Relationship between Drugs and Diseases

In this work, disease-related genes were taken as the starting point of random walk on one side, and the target genes of drugs were taken as the starting point of random walk on the other side. Through the restart random walk on the whole PPI network, the relationship between each disease and each drug on the PPI network was obtained, and their correlation coefficient was further calculated. We got 18564 group correlations of 78 diseases and 238 drugs. According to their correlation coefficients, 61 pairs of disease drugs with a correlation degree of more than 0.8 are found, of which 53 diseases and drugs have been confirmed by research, and 8 pairs belong to unknown drug-disease relationship. The relevant information of 8 pairs of diseases and drugs is shown in Table 2.

Methylprednisolone (DB00959) can treat autoimmune diseases, but we found that methylprednisolone is strongly associated with hematological diseases. According to the definition of MeSH, blood diseases include blood tumors, bone marrow diseases, and other diseases. Methylprednisolone is a biological macromolecular drug, a steroid derivative, and also a glucocorticoid. It can affect the expression of some genes through the cell membrane, thus interfering with the inflammatory response, inhibiting humoral immune response, and has a strong anti-inflammatory effect. Bowen et al. found that high-dose methylprednisolone has a certain effect on patients with recurrent chronic lymphoblastic leukemia [27]. Yao et al. found that methylprednisolone inhibited Wnt signaling pathway by downregulating the expression of LEF-1 protein, and Wnt signaling pathway is highly related to recurrent chronic lymphoblastic leukemia [28].

Mitoxantrone (DB01204) is associated with non-Hodgkin's lymphoma (NHL) and multiple sclerosis (MS). We found that it is also strongly correlated with lymphoid leukemia [29, 30]. Mitoxantrone has significant benefits for tumor control and overall survival in patients with recurrent acute lymphoblastic leukemia.

Prednisolone (DB00860) is a typical steroid drug, which can treat a variety of diseases, including rheumatoid arthritis, asthma, allergies, psoriasis, and multiple sclerosis [31]. However, these diseases are all autoimmune diseases. Therefore, we also found that prednisolone has a strong connection with autoimmune diseases.

We also found that apomorphine (DB00714), cabergoline (DB00248), bromocriptine (DB01200), and rotigotine (DB05271) are related to Parkinson's disease. After querying DrugBank, we knew that these four drugs have therapeutic effects on Parkinson's disease, but they are not included in the known data set.

### 3.3. GO Function Enrichment Analysis

Eight reusable drugs were found in this work, five of which have pharmacodynamic effects on Parkinson's diseases. We further performed GO function enrichment analysis on disease-related genes of the disease before drug action. The results are shown in Figure 2(a). It is easy to note that genes are mainly enriched in functional modules such as chromosome breakage (GO: 0031052), upregulated cell migration (GO:0030335), and chain replacement (GO:0000732).

We then analyzed the related genes of Parkinson's diseases after drug action. The results are shown in Figure 2(b). The results show that the gene is enriched in the following functional modules, such as the regulation of exercise (GO:0040012), dopamine binding (GO:0035240), and serotonin binding (GO:0051378).

Before and after random walk, the GO enrichment module of Parkinson's disease has changed significantly. Before random walk, the main enrichment module of Parkinson's syndrome is related to gene expression and cell movement in cells, which may be related to the pathogenesis of Parkinson's disease. After random walk, the relevant genes of Parkinson's syndrome are mainly enriched in some neural transmission modules, which are closely related to the treatment of Parkinson's syndrome.

### 3.4. KEGG Pathway Analysis

We further analyzed the genes related to Parkinson's disease by KEGG pathway. The results are shown in Figure 3.  Figure 3(a) shows that genes are mainly enriched in pancreatic secretion (hsa04972), PI3K Akt signaling pathway (hsa04151), and other pathways. After adding drug information and random walk, we conducted KEGG pathway analysis on relevant genes. The results show that the genes are mainly enriched in neural active ligand receptor interaction (hsa04080), calcium signaling pathway (hsa04020), serotonin receptor synapse (hsa04726), and dopamine receptor synapse (hsa04728).

Before and after random walk, the KEGG pathway enrichment module of Parkinson's disease has changed significantly. The approximate change is similar to the result of GO enrichment analysis. Before random walk, the main enrichment pathways of Parkinson's syndrome are related to intracellular signaling pathways. After random walk, the relevant genes of Parkinson's syndrome are mainly enriched in some neural transmission pathways, which are closely related to the treatment of Parkinson's syndrome.

### 3.5. Key Gene Analysis

In order to further study key genes of Parkinson's disease, we studied the local relationship between Parkinson's disease and trihexyphenidyl, a drug that can treat Parkinson's disease and their related genes on the network (Figure 4). It can be seen from Figure 4 that the key genes of Parkinson's disease are *α*-synuclein (Gene ID: 6622) and tau protein (Gene ID:4137). *α*-Synuclein mainly exists at the synapse of the nerve cells and plays a key role in the transmission of neurotransmitters. Tau protein is a microtubule-associated protein that mainly exists in nerve cells. These two proteins are closely related to the pathogenesis of Parkinson's disease.

## 4. Conclusion

With the prevalence of complex diseases, the existing drugs are far from meeting the needs of human beings to fight diseases. At the same time, due to the rising cost of drug research and development and the long research and development cycle, the research and development means of innovative drugs have become a major challenge in the medical field. In recent years, with the continuous enrichment of disease and drug databases, researchers have realized drug reuse through the correlation analysis of disease-related genes, drugs, and drug-target data. This is a new research and development idea in the field of pharmaceutical research and development, which reduces the research and development cost of innovative drugs and saves resources. Because most diseases are not single gene defects, they often involve the destruction of the coordination function between genes [32]. Therefore, we explored the relationship between drugs and diseases based on the biological function network. Using HPRD, BioGRID, STRING, and other databases; the protein–protein interaction (PPI) network was constructed. We designed a combination algorithm of random walk and supervised learning to predict the sensitivity of drugs. The accuracy of sensitivity prediction is 82.7%.

With the help of the proposed method, we found that 8 pairs of drug-disease relationships have not been reported, and 5 of them have pharmacodynamic effects on Parkinson's diseases. For Parkinson's disease, we found the changes of its functional modules by adding drug information and comparing before and after random walk, combined with the results of GO and KEGG function enrichment analysis. Using the network diagram of disease and drug-related genes after random walk, we found the key linkage between Parkinson's disease and phenylhexol, a drug for the treatment of Parkinson's disease *α*-synuclein and tau protein, which provide a useful exploration for the effectiveness of the treatment of Parkinson's disease.

## Figures and Tables

**Figure 1:** The AUC distribution of the random walk with restart method and supervised learning.

**Figure 2:** The distribution of the related genes of Parkinson's diseases. (a) GO function enrichment on the disease-related genes of Parkinson's disease before drug action; (b) GO function enrichment on disease-related genes of Parkinson's disease after drug action.

**Figure 3:** KEGG pathway of the related genes of Parkinson's diseases. (a) KEGG pathway on the disease-related genes of Parkinson's disease before drug action; (b) KEGG pathway on disease-related genes of Parkinson's disease after drug action.

**Figure 4:** The gene network between Parkinson's disease and trihexyphenidyl.

**Table 1:** Average AUC value of various diseases based on the random walk with restart method and three PPI networks BioGrid, HPRD, and STRING.

Disease classification based on MeSH	Number of diseases	Average AUC
Viral diseases C02	2	0.70467
Tumor C04	16	0.764632
Musculoskeletal diseases C05	5	0.748488
Digestive system diseases C06	9	0.760698
Respiratory diseases C08	2	0.68288
Nervous system diseases C10	9	0.62232
Eye diseases C11	2	0.83772
Male genitourinary system C12	1	0.81407
Cardiovascular disease C14	11	0.66685
Blood and lymphatic system C15	4	0.876637
Skin and connective tissue diseases C17	5	0.675556
Nutritional and metabolic diseases C18	6	0.734407
Endocrine system diseases C19	2	0.87446
Immune system diseases C20	4	0.62869

**Table 2:** The relevant information of eight diseases and eight drugs.

Disease	Drug	Pearson
Parkinsonian disorders	Apomorphine	0.876
Parkinsonian disorders	Cabergoline	0.876
Bone diseases metabolic	Calcitriol	0.841
Parkinsonian disorders	Bromocriptine	0.840
Leukemia lymphoid	Mitoxantrone	0.834
Hematologic diseases	Methylprednisolone	0.811
Parkinsonian disorders	Rotigotine	0.806
Autoimmune diseases	Prednisolone	0.806

## Data Availability

The data used to support the findings of this study are available from the Protein–Protein Interaction (PPI) Network: https://ppi-net.org
